# Epigenetic Silencing of Peroxisome Proliferator-Activated Receptor γ Is a Biomarker for Colorectal Cancer Progression and Adverse Patients' Outcome

**DOI:** 10.1371/journal.pone.0014229

**Published:** 2010-12-03

**Authors:** Massimo Pancione, Lina Sabatino, Alessandra Fucci, Vincenzo Carafa, Angela Nebbioso, Nicola Forte, Antonio Febbraro, Domenico Parente, Concetta Ambrosino, Nicola Normanno, Lucia Altucci, Vittorio Colantuoni

**Affiliations:** 1 Department of Biological and Environmental Sciences, University of Sannio, Benevento, Italy; 2 Department of General Pathology, Second University of Naples, Napoli, Italy; 3 CNR-IGB, Napoli, Italy; 4 Departments of Medical Oncology and Clinical Pathology, Fatebenefratelli Hospital, Benevento, Italy; 5 Biogem “G. Salvatore” Genetic Research Institute, Ariano Irpino, Italy; 6 Pharmacogenomic Laboratory, Center for Oncology Research, Mercogliano, Italy; University of Hong Kong, Hong Kong

## Abstract

The relationship between peroxisome proliferator-activated receptor γ (*PPARG*) expression and epigenetic changes occurring in colorectal-cancer pathogenesis is largely unknown. We investigated whether *PPARG* is epigenetically regulated in colorectal cancer (CRC) progression. *PPARG* expression was assessed in CRC tissues and paired normal mucosa by western blot and immunohistochemistry and related to patients' clinicopathological parameters and survival. *PPARG* promoter methylation was analyzed by methylation-specific-PCR and bisulphite sequencing. *PPARG* expression and promoter methylation were similarly examined also in CRC derived cell lines. Chromatin immunoprecipitation in basal conditions and after epigenetic treatment was performed along with knocking-down experiments of putative regulatory factors. Gene expression was monitored by immunoblotting and functional assays of cell proliferation and invasiveness. Methylation on a specific region of the promoter is strongly correlated with *PPARG* lack of expression in 30% of primary CRCs and with patients' poor prognosis. Remarkably, the same methylation pattern is found in *PPARG*-negative CRC cell lines. Epigenetic treatment with 5′-aza-2′-deoxycytidine can revert this condition and, in combination with trichostatin A, dramatically re-activates gene transcription and receptor activity. Transcriptional silencing is due to the recruitment of MeCP2, HDAC1 and EZH2 that impart repressive chromatin signatures determining an increased cell proliferative and invasive potential, features that can experimentally be reverted. Our findings provide a novel mechanistic insight into epigenetic silencing of *PPARG* in CRC that may be relevant as a prognostic marker of tumor progression.

## Introduction

Peroxisome Proliferator-Activated Receptors (PPARs) are ligand-dependent transcription factors belonging to the nuclear hormone receptor superfamily [1]. Three different PPAR isoforms, α, β and γ have been isolated so far, each with a distinct pattern of tissue expression and ability to interact with diverse classes of compounds. Specifically, the PPARγ isoform is implicated in a wide range of physiological processes [2]: it integrates the control of energy, lipid and glucose homeostasis and plays a pivotal role in adipogenesis, inflammatory response and differentiation of many epithelial cells [3]. Consistently, variations in *PPARG* expression or gene mutations have been associated with tumorigenesis [4]–[6]. However, conflicting results have been reported so far, raising the question as to whether PPARγ facilitates or suppresses tumorigenesis [7], [8]. Recently, we have shown that sporadic colorectal cancers (CRCs) presenting reduced PPARγ expression levels are significantly associated with patients' worse prognosis; in the same type of tumours, *PPARG* has been shown to be an independent prognostic factor [9], [10], suggesting the possibility to target this gene with drugs in clinical applications [10]. The molecular mechanisms underlying *PPARG* expression regulation in CRC progression are still unknown [9].

It is becoming increasingly clear that, in addition to genetic alterations, epigenetic modifications contribute to tumorigenesis [11]. Epigenetic regulation involves heritable modifications that do not change the DNA sequences but provide “extra” layers of control to regulate chromatin organization and gene expression [12]. Aberrant DNA methylation at CpG-rich sequences, also known as “CpG islands”, located in the promoter regions of approximately half of the known genes, leads to epigenetic silencing of gene expression [11], [12]. In CRC, extensive DNA methylation has been detected at several loci, specifically at the promoter regions of tumor suppressor genes (TSG), a characteristic of a subgroup of tumours presenting the so-called “CpG island methylator phenotype” (CIMP) [13]. Other epigenetic events, such as repressive histone modifications, cooperate to establish stable gene silencing. A “histone code” has been suggested to provide a signature on specific amino acid residues that correlates with active or repressed gene expression [11], [12]. The link between DNA methylation and histone modifications seems to be mediated by Methyl CpG DNA binding proteins, a member of which MeCP2 plays an important role to establish this interaction [14]. DNA methylated regions, usually enriched in modified histones, generate a more tightly packed chromatin where the access of specific transcription factors to their cognate binding sites is greatly impaired [12]. How DNA methylation and the pattern of histone modifications on promoter regions of specific genes are associated with cancer initiation and progression, in particular in sporadic CRC, remains to be elucidated [15]. In this report, we analyzed one-hundred and fifty-two primary CRCs and paired normal mucosa in order to correlate *PPARG* expression variations mediated by epigenetic events with tumor progression and patients' survival. We extended the analysis to CRC derived cell lines as a system to investigate the molecular mechanisms underlying *PPARG* silencing due to epigenetic variations.

## Materials and Methods

### Ethics Statement

This study was conducted according to the principles expressed in the Declaration of Helsinki. The study was approved by the Institutional Review Board of Fatebenefratelli Hospital in Benevento. All patients provided written informed consent for the collection of samples and subsequent analysis.

### Tumor samples

One hundred and fifty-two patients diagnosed primary sporadic CRC and surgically treated at the Department of Surgery, Fatebenefratelli Hospital, Benevento, Italy, between 1999–2004, were investigated in this study. Fifty-two cases comprise both liquid nitrogen snap-frozen specimens, obtained immediately after surgical resection, and paraffin blocks. Each sample was matched with the adjacent apparently normal mucosa (at 20 cm distance from the tumor mass) removed during the same surgery. None of the patients had a familial history of intestinal dysfunction or CRC, had received chemotherapy or radiation prior to resection nor had taken non steroidal anti-inflammatory drugs on a regular basis. Conventional postoperative treatments were provided to all patients, depending upon the severity of the disease. The clinico-pathological features of the patients investigated are reported (**Table 1**). The follow-up was available for all patients, with a median post-operative duration of 59.5±26.5 months. Overall length of survival was calculated starting from the first surgery. Patients were prospectively followed until death or their most recent medical examination.

**Table 1:** Correlation between *PPARG* promoter methylation and several clinico- pathological parameters of the patients.

*Parameters*	N	M3 PPARG methylation		P
		Met	Umet	
*Gender*				0.719
Male	95	31	64	
Female	57	17	40	
*Age(Years)*				0.001**
≤60	32	18	14	
>60	120	30	90	
*Location* a				0.230
Proximal	56	21	35	
Distal	96	27	69	
*Tumor size*				0.683
≤5 cm	51	15	36	
>5 cm	101	33	68	
*Differentiation*				0.069
Well/Mod	129	37	92	
Por	23	11	12	
*Histology* b				0.110
AD	123	36	87	
AD-MUC	26	10	16	
MUC	3	2	1	
*T stage*				0.05*
pT1	9	2	7	
pT2	12	5	7	
pT3	125	37	88	
pT4	6	4	2	
*N stage*				0.002**
N0	111	26	85	
N1	25	14	11	
N2	16	8	8	
*Distant Metastasis*				0.0001**
M0	107	23	84	
M1	45	25	20	
**Total**	**152**	**48**	**104**	

a Proximal: caecum, ascending and transverse colon; Distal: descending and sigmoid colon, rectum;

b AD  =  adenocarcinoma; AD-MUC =  adenocarcinoma with a mucinous component below 50%; MUC =  adenocarcinoma with a mucinous component above 50%. Abbreviations: Well = well-differentiated; Mod = moderately differentiated; Por = poorly differentiated adenocarcinoma. χ^2^ test;

*Significant at 0.05 level;

**Significant at 0.01 level. Patients' mean age was 71.1±12.3 years old. The classification of the tumours was based on the TNM (Tumor-Node-Metastasis) system according to the criteria of the International Union Against Cancer (UICC).

### Cell lines and 5′-aza-2′-deoxycytidine and Trichostatin A treatment

Twelve CRC derived cell lines were used in this study and were obtained from the ATCC and cultured as suggested. For DNA demethylation, cells were treated with 1 or 5 µM 5′-aza-2′-deoxycytidine (AZA) for 72 hs or 300 nM Trichostatin A (TSA) (Sigma-Aldrich, St. Louis, USA) for 24 hs, alone or in combination. After the treatments, cells were harvested for DNA, RNA or protein extraction.

### DNA extraction, bisulphite treatment, methylation analysis and sequencing

Genomic DNA was isolated from frozen tissues or from paraffin embedded samples using a standard procedure [6], or the FFPE tissue kit (56404, Qiagen, Hilden, Germany), respectively. One µg of each DNA sample was bisulphite modified according to the manufacturer's protocol (59104, Qiagen, Hilden, Germany). Both universally unmethylated (59665) and CpGenome universally methylated DNA (59655, Qiagen, Hilden, Germany) were used in each reaction as unmethylated or methylated control, respectively. The search for CpG content in the *PPARG* promoter was performed using the Methprimer software according to CpG island definition. PCR primers for methylation specific PCR (MS-PCR) were designed using Methyl Primer Express software v1. Both unmethylated (U) and methylated (M) specific sets of primers were designed based on the positive strand of the bisulfite-converted DNA covering the CpG islands within the *PPARG* promoter region. MS-PCR reactions were performed using the MS-PCR kit (59305, Qiagen, Hilden, Germany) following the manufacturer's instructions. PCR products were loaded onto non-denaturing 3% agarose gels, stained with ethidium bromide, and visualized under an UV transilluminator. Primer sequences are listed (**Table S1**). Bisulphite sequencing (BS) was automatically carried out on the PCR amplification product obtained by using a primer set not containing CpG sites within their sequences and designed on bisulphite modified DNA (Applied Biosystems, Applera, Foster City, USA).

### ChIP and MeDIP assay

ChIP assays and q-PCR amplification (Biorad, Hercules, USA) were performed as described [16]. The primers used are described (**Table S1**). MeDIP assay was carried out as recommended by the supplier (Diagenode, Liège, Belgium). Antibodies raised against: AcH3K9, H3K4me3, HDAC1 and MeCP2 (Abcam, Cambridge, UK), H3K27me3, (Millipore, Billerica, USA), RNA pol II and P-RNA pol II (Covance, Dallas, USA), ZAC and purified IgG (Santa Cruz Biotechnology, Santa Cruz, USA) were used in ChIP assays.

### Western blot and immunohistochemical analysis

Western blot analysis was performed on protein extracts from tumor tissues and adjacent normal mucosa taken during surgery and CRC cell lines, as previously reported [6], [9]. Immunohistochemical analysis on tumors and distant non-neoplastic mucosa was performed as described [9]. The following antibodies were used: anti-PPARγ (E-8), anti-ZAC (H-253), anti-ERK 1/2 (MK1) and anti-p-ERK (E-4) (Santa Cruz Biotechnology, Santa Cruz, USA); anti-E-cadherin (610405) (BD Transduction Laboratories, Lexington, USA); anti-MeCP2 (ab55538), anti-HDAC1 (ab19845) (Abcam, Cambridge, UK); anti-EZH2 (4905) (Cell Signaling, Boston, USA); anti-β-actin (A5441) (Sigma-Aldrich, St. Louis, USA).

### MTT and apoptosis assays

Cells were seeded in triplicate in 24 or 96 well-plates and the MTT assay (Sigma-Aldrich, St. Louis, USA) was performed according to the manufacturer's protocol at 0, 24, 48, 72 and 96 hs after reaching confluence, as indicated. The growth curves were set up taking into account the average results obtained from three independent experiments. To analyze chemo-sensitivity to PPARγ agonists cells were treated with 5 µM troglitazone (TZD). Apoptosis assay was performed by flow cytometric analysis (FCA) using propidium iodide (PI) staining. Briefly, after incubation with TZD, cells were harvested and fixed in 70% ice-cold ethanol/PBS and stored at 4°C overnight. The suspended cells were then washed with PBS, incubated in a PI solution for 15 min. at 37°C and immediately analyzed with a FAC scan flow cytometer (Becton Dichinson, San Jose, USA).

### Migration and invasion assays

For the wound-healing assay, cells were plated in 60-mm plates and grown to confluence. After a 6 hs long serum starvation, a wound was made by using a micropipette tip to scrape off the cells. Cell motility was studied after 24 and 48 hs, following cells from different microscope fields. Finally, the corresponding wound area at each time point was digitalized and quantified using Metamorph Imaging System Software version 6.0 for Microsoft Windows. An average percentage of wound closure was calculated from three independent experiments. To determine invasiveness a transwell assay was carried out using a 24 well cell culture insert, 8 µm pore (3097, Falcon-Becton Dickinson, USA). Following hydration of the matrigel in the upper compartment, cells were seeded and incubated. Twenty-four and forty-eight hs later the cells of the upper surface of the filter were removed with a cotton swab; those underneath were fixed with 4% paraformaldehyde, stained with 0,2% crystal violet and counted. Quantification was obtained by counting at least 10 lower power fields from three independent experiments.

### RNA extraction and semi-quantitative reverse transcription-PCR

Total RNA was isolated from cell lines and tissues with Trizol with minor modifications (Invitrogen Carlsbad, USA). Reverse transcription-PCR (RT-PCR) was made using Super-script II (Invitrogen, Carlsbad, USA) and PCR amplification using specific primers for *PPARG*. The RT-PCR conditions and the primers used have previously been reported [5]. In all PCR reactions, *GAPDH* served as an internal control for normalization. The amplified products were run on a 2% agarose gel and stained with ethidium bromide.

### Plasmids and transfections

The PPRE-TK driven luciferase reporter plasmid, the pcDNA3 carrying the wild type *PPARG* cDNA and the transfection conditions have already been described [6]. For gene re-activation assays, cells were seeded in 6-well plates, treated with AZA and TSA alone or in combination and transiently transfected with the reporter plasmid. After 12 hs, 1 µM TZD or the vehicle alone were added to the medium. When indicated, GW9662, a selective PPARγ antagonist, was used.

### siRNA

A retroviral vector PSM2C (clone ID VH2-203345) that carries a short hairpin DNA (shRNA, catalog number RHS1764-9494331) for targeting PPARγ mRNA was used. HT29 cells were stably transfected with the shRNA-PPARγ vector and the positive clones selected by using 1 µM puromycin. A vector carrying non-specific shRNAs or an empty vector were used as controls. The siRNA designed for targeting human MeCP2 mRNA (code: HS-MECP2-7HP SI02664893, Qiagen, Hilden, Germany) was kindly provided by Prof. Chiariotti. HCT116 cells were seeded in 6-well plates and transiently transfected with the MeCP2 siRNA or non-specific oligos, according to the manufacturer's instructions (Invitrogen, Carlsbad, USA). To silence EZH2, a retroviral vector PSM2C carrying an EZH2-shRNA (code: RHS1764-9100483, CN: V2HS-63033) scrambled shRNAs or an empty vector were used, according to the manufacturer's instructions (Invitrogen, Carlsbad, USA). In both cases, cells were harvested for western blot analysis 56 hs later.

### Loss of heterozygosity, *BRAF* and *KRAS* mutations and microsatellite instability analysis

Loss of heterozygosity (LOH) was assessed as previously described, using the microsatellite markers D31259 and D3S3701, which flank *PPARG* [6]. Microsatellite instability (MSI) was performed as reported [17]. *MLH1* promoter methylation was also assessed on some representative tumour samples [18]. *BRAF* and *KRAS* mutations at codon 600 in exon 15 and codons 12/13 in exon 2, respectively, were evaluated by PCR/sequencing and Real-Time PCR using primers previously described [18].

### Statistical analysis

All statistical analyses were carried out with the SPSS (version 15.0) for Windows (SPSS Inc., Chicago, USA). Association between *PPARG* promoter methylation, other markers and clinico-pathological parameters was assessed using the χ^2^ test or the Spearman rank test, as indicated. The Kaplan-Meier method was used to estimate survival; survival differences were analyzed with the log-rank test. Data were reported as mean ± SD, and mean values were compared using the Student's t test or Mann-Whitney test. Results were considered statistically significant when a *P*≤0.05 was obtained.

## Results

### *PPARG* promoter methylation in CRCs correlates with gene expression and is associated with patients' outcome

To assess the role that *PPARG* plays in colorectal tumorigenesis *in vivo*, we analyzed 152 primary sporadic CRCs and the matched adjacent non-neoplastic mucosa for *PPARG* expression (**Figure 1** **, panel A**). About 60% of tumors showed *PPARG* over-expression and 5% of cases showed not significant differences between tumour tissues and the matched normal mucosa. In contrast, 35% of the tumours showed lower PPARγ levels than the normal mucosa and a significant association with distant metastases and reduced patients' survival, in line with our previous data (**Figure 1** **, panels B and C**) [9]. We have already reported that reduced *PPARG* expression in sporadic CRCs is not associated with LOH [6]. Thus, to determine whether *PPARG* reduced expression is correlated with DNA methylation, we examined the entire promoter region. Inspection of the human *PPARG* promoter showed that the core region, from −474 to +600 with respect to the transcription start site, is particularly enriched in “CpG islands” that might be target of DNA methylation (**Figure 1** **, panel D**). A shorter CpG-rich DNA tract located upstream (from −793 to −580) has been found stably methylated in a study evaluating the epigenetic risk factor associated with the early onset of adult metabolic syndrome (**Figure 1** **, panel D**) [19]. To investigate whether these two regions are differentially methylated in primary CRCs and paired normal mucosa, we performed MS-PCR on four promoter segments (M1 to M4 starting from the more downstream) (**Figure 1** **, panel D**). Segments M4 (from−746 to −616) and M1 (from −123 to +49) were always methylated or unmethylated in normal and tumor samples and were not correlated with *PPARG* expression levels (**Figure 1** **, panel E**). M2 (from −235 to −151) was variably methylated and, finally, M3 (from −359 to −260) was methylated in about 30% of tumours as compared to 8% of paired normal mucosas (n = 80) and correlated with reduction/loss of *PPARG* expression (**Figure 1** **, panel E and** **Table 1**). A closer inspection of the M3 segment identified 9 CpG sites, the methylation status of which was analyzed by bisulphite sequencing (**Figure 1** **, panel F**). The CpG islands methylation level was significantly higher in *PPARG*-negative than *PPARG*-positive tumours and paired normal mucosas (**Figure 1** **, panel G**). Consistently, the M3 region methylation correlated with patient's age, deep invasion, Duke's C and D stages, whereas no association was detected with tumour location (proximal or distal colon) and gender (**Figure 1** **, panel H and** **Table 1**). *PPARG* methylation was more frequently observed in a subgroup of microsatellite high (MSI-H) than in microsatellite stable (MSS) tumours. Moreover, these cases were not related with *KRAS* or *BRAF* mutations (**Figure S1**). All together these results indicate that *PPARG* promoter methylation, specifically at the M3 region, is significantly correlated with tumour progression and patients' poor outcome (**Figure 1** **, panel I**).

**Figure 1:** A specific *PPARG* promoter methylation is associated with protein expression and patients' poor prognosis. (**A**) Fifty µg of total protein extracts from tumour tissues (T) and matched non-neoplastic mucosa (N) were analyzed by Western blot. In the panel only some representative samples (from 1 to 8) are shown. The histogram reports the quantification to β-actin, used as internal control. (**B**) Correlation of *PPARG* expression levels in the absence = M0 or presence = M1 of distant metastases. (**C**) Kaplan Meier survival analysis related to *PPARG* expression levels. The *P* value is reported in each graph. (**D**) Schematic structure of the *PPARG* promoter and identification of the CpG-enriched regions encompassing the transcription start site of the human gene. The MS-PCR regions analyzed (M1–M4) and the positions of the primers used are depicted as rectangles. (**E**) Representative MS-PCRs show a correlation between methylation of the M3 region and reduced *PPARG* expression in tumour tissues vs. matched normal mucosa, C+ indicates methylated (M) and unmethylated (U) controls. (**F**) The M3 nucleotide sequence is reported; the CpG islands are highlighted. The chromatograms show which CpG dinucleotide is methylated in some representative samples after BS. Black or white circles indicate the methylated or unmethylated cytosines, respectively. (**G**) Methylation levels detected by BS in tumour and normal mucosa specimens. The M3 region methylation is related to tumour' stage (Duke's from A to D) (**H**) and patients' survival (**I**). The *P* value is reported in each graph.

### *PPARG* silencing in CRC cell lines correlates with promoter methylation

To investigate the molecular mechanism(s) underlying this relationship, we sought to use an *in vitro* cell culture system. We screened a series of human CRC cell lines (**Table S2**) for *PPARG* expression levels and correlated these with possible silencing events. PPARγ expression was investigated at the mRNA and protein level by RT-PCR and western blot analysis, respectively (**Figure 2** **, panel A**). PPARγ mRNA mirrored protein levels with a wide range of variations from the highest in HT29 to the lowest in HCT116 cells. The differences detected were attributed to transcription variations; a reduced protein expression not related to mRNA levels was observed only in Caco-2 cells, likely due to post-translational mechanism(s). Among these cell lines, we selected HT29 and HCT116 for further investigations. We did not detect loss of heterozygosity at the *PPARG* locus in both cell lines. Similarly, we did not correlate the different *PPARG* levels observed in HCT116 and HT29 cells with post-translational modifications caused by an active mitogen-activated protein kinase (MAPK/ERK) pathway (**Figure S2**) [6], [20]. To investigate whether *PPARG* expression correlates with promoter methylation in the CRC cell lines, we performed MS-PCR (**Figure 2** **, panel B**). The M4 and M1 segments were stably methylated or unmethylated in all cell lines, regardless of PPARγ expression. The M2 segment was methylated in 5 out of 8 cell lines, including HCT116. Interestingly, the M3 segment was methylated only in HCT116 out of the eight CRC cell lines analyzed (**Figure 2** **, panel B**). By examining four additional CRC cell lines, we found that also RKO cells were negative for *PPARG* expression, due to aberrantly methylated M3 region (**Table S2 and data not shown**). MeDIP assays confirmed these results: the *PPARG* promoter DNA (from −368 to −166) was three-fold more methylated in HCT116 than in HT29 cells, indicating a more tightly packed chromatin structure (**Figure S2**). 90% of the CpG sites contained in the M3 segment were methylated in HCT116, whereas only few or none were methylated in other cell lines as assessed by bisulphite sequencing (**Figure 2** **, panel C**). These findings suggest that promoter methylation could play a role in silencing *PPARG* expression in the CRC cell lines analyzed.

**Figure 2:** Promoter methylation is associated with reduced *PPARG* expression levels in CRC cell lines. (**A**) *PPARG* mRNA and protein levels detected by RT-PCR ad western blot analysis in a panel of eight CRC cell lines. *GAPDH* and β-actin were used as controls, respectively. (**B**) MS-PCR results obtained on the M1–M4 promoter regions analyzed; M, methylated; U, unmethylated; C+ indicates methylated and unmethylated controls. The methylation status of all CRC cell lines analyzed is summarized, with HCT116 and HT29 cells depicted in grey. (**C**) CpG dinucleotides methylation was assessed by BS. The results of some representative cell lines are reported. Methylated or unmethylated CpG dinucleotides are depicted as black or white circles, respectively. (**D**) Pharmacologic demethylation induced *PPARG* expression in HCT116 while no significant difference was found in HT29 cells used as control. Cells were exposed to 1 and 5 µM AZA for 72 hs, MS-PCR was carried out on the M2 and M3 regions, before and after treatment, **P<0.01.

### *PPARG* expression is re-activated by pharmacologic demethylation

To verify whether *PPARG* expression can be re-activated by pharmacologic demethylation, we treated HCT116 cells with AZA, a well-known inhibitor of DNA methylation. RT-PCR analysis from HCT116 exposed to 1 and 5 µM AZA showed a dose-dependent increase of the PPARγ mRNA whereas did not show significant variations in HT29 cells, as expected (**Figure 2** **, panel D**). MS-PCR performed on the M3 region, that is methylated only in HCT116 cells, showed loss of methylation following the treatment; the M2 region, that in basal conditions is methylated in both cell lines, got demethylated after the treatment (**Figure 2** **, panel D**). All together these data demonstrate that extensive promoter methylation is associated with reduced *PPARG* expression in CRC cell lines.

### Co-operative effect of AZA and TSA on *PPARG* re-activation

That specific regions of the *PPARG* promoter are differentially methylated points out that epigenetic mechanism(s) are involved in its deregulated expression in CRC cells. To verify this hypothesis, we treated HCT116 with AZA, alone or in combination with TSA, a known histone deacetylase inhibitor (HDACi). HT29 cells were used as a control. *PPARG* expression was synergistically induced by the combined treatment with AZA and TSA in HCT116 cells while was not affected in HT29 cells, when the drugs were used either alone or in combination (**Figure S3**). These data indicate that chromatin-associated histone enzymes may contribute to gene silencing. To determine whether the re-activated PPARγ behaves as a *bona fide* functional transcriptional factor, we treated HCT116 cells with AZA or TSA alone or in combination and subsequently transfected with a PPRE-driven luciferase reporter gene. Luciferase activity determined in cell extracts increased upon AZA and/or TSA treatment and, strikingly, even further upon addition of troglitazone, a specific PPARγ ligand (**Figure S3**). To demonstrate that the increase in luciferase activity was really dependent upon the re-activated receptor, we exposed the transfected cells to the PPARγ antagonist, GW9662. A significant reduction of reporter gene activity was observed due to GW9662 ability to irreversibly interfere with the transactivating ability of the mature protein (**Figure S3**). All together these data show that DNA promoter methylation and histone modifications likely co-operate to down-regulate *PPARG* expression, suggesting that epigenetic treatments re-establish gene transcription and activity.

### Specific repressive chromatin marks and DNA methylation are associated with *PPARG* transcription

To provide insights into the mechanism(s) by which DNA methylation and histone modifications affect *PPARG* expression, quantitative ChIP assays were performed investigating the promoter segment extending from −368 to −166 in HCT116 cells. Consistent with the MeDIP data, HDAC1 was tightly bound to *PPARG* promoter, whereas RNA-Polymerase II (RNAPol-II) and its phosphorylated form (P-RNAPol-II) were barely present in untreated HCT116 cells (**Figure 3** **, panel A**). Upon exposure to AZA and TSA in combination, HDAC1 was remarkably depleted along with a reduced DNA methylation (**Figure S2**), whereas RNAPol-II and P-RNAPol-II were greatly enhanced, indicating transcription recovering (**Figure 3** **, panel A**). Accordingly, trimethylated H3K4 and acetylated H3K9, that are histone modifications normally associated with transcriptional activity, were almost reduced in untreated HCT116 cells and significantly increased with TSA, AZA or their combination (**Figure 3** **, panel B**). Of note, trimethylated H3K9, a marker of silenced chromatin, was enriched at the *PPARG* promoter and progressively depleted after epigenetic treatments, while trimethylated H3K27 was significantly reduced only by the AZA/TSA combined treatment (**Figure 3** **, panel C**). This analysis suggests that DNA methylation is closely associated with repressive chromatin marks at the *PPARG* promoter to impair gene expression in CRC cells.

**Figure 3:** *PPARG* transcriptional repression is due to specific repressive chromatin marks and recruitment of HDAC1. (**A**) Quantitative ChIP analysis in HCT116 cells was performed before and after the treatment with AZA and TSA alone or in combination. Native chromatin was incubated with antibodies directed against the indicated proteins. The immunoprecipitated DNA was used as template in qPCR reactions using specific primers for the *PPARG* promoter region *P<0.05, **P<0.01. (**B**) ChIP assays were carried out as described above against acetylated H3K9 and trimethylated H3K4 *P<0.05, **P<0.01 or (**C**) trimethylated H3K9 and H3K27 *P<0.05. The time-points for co-treatments were 72 hs for 5 µM AZA and 24 hs for 300 nM TSA, alone or in combination; CC indicates untreated control cells. Results are the mean values ± SD of three independent experiments, each performed in duplicate.

### siRNA mediated knock-down of MeCP2 and EZH2 rescues *PPARG* expression in HCT116 colon cancer cells

The link between DNA methylation and histone modifications appears to be mediated by a group of proteins with methyl DNA binding activity that includes methyl CpG binding protein 2 (MeCP2) [14]. These proteins localize to methylated promoter regions and recruit protein complexes containing HDACs, especially HDAC1, and histone methyltransferases (HMTs). Enhancer of zeste 2 (EZH2) is a member of the polycomb repressor complex 2 (PRC2) with histone methyl-transferase activity at specific H3K27 sites [21]. Both MeCP2 and EZH2 have been reported to be involved in *Pparg* repression in mouse stellate cells undergoing liver fibrogenesis [22]. *PPARG* transcriptional activation, on the other hand, appears to be modulated by the zinc-finger protein (ZAC) likely together with other still unknown factors [23]. MeCP2, EZH2 and HDAC1 were more expressed in HCT116 than HT29 cells, thus inversely correlating with PPARγ, whereas ZAC levels directly associated with PPARγ (**Figure 4** **, panels A and B and Figure S4**). In line with this, ChIP analysis showed that ZAC was more recruited in HT29 than HCT116 cells. (**Figure 4** **, panel B**). Importantly, in *PPARG*-negative cells following epigenetic treatment, ZAC became highly enriched at the promoter correlating with *PPARG* transcription recovery (**Figure 4** **, panel B**). ChIP assays performed in the same setting showed that MeCP2 was highly recruited at the *PPARG* promoter in basal conditions and depleted after treatment with AZA or TSA alone or in combination (**Figure 4** **, panel C**). Accordingly, silencing MeCP2 caused a marked increase of *PPARG* expression (**Figure 4** **, panel D**). In the same HTC116 cells, the *PPARG* promoter was particularly enriched in H3K27me3 (**Figure 4** **, panel E**). Knocking-down EZH2 associated with a three-fold increase of PPARγ and reduction of H3K27me3 at the *PPARG* promoter as compared with control cells (**Figure 4** **, panel F**). Finally, MeCP2, HDAC1 and EZH2 levels were examined in a subset of CRCs. HDAC1 and EZH2 levels were more expressed in tumour tissues than the paired normal mucosas and directly correlated with advanced Duke's stages (**Figure S4**). MeCP2, in contrast, was unchanged or slightly increased in the same subset of tumours (**Figure S4**). Altogether these results indicate that MeCP2, HDAC1 and EZH2 are involved in *PPARG* repression in colon tumorigenesis both *in vivo* and *in vitro*.

**Figure 4:** MeCP2 and EZH2 are negative regulators of *PPARG* expression in CRC cell lines. (**A**) Western-blot analysis shows higher levels of MeCP2 and EZH2 in HCT116 than HT29 cells *P<0.01. (**B**) In contrast, ZAC is more expressed in HT29 than HCT116 cells, thus directly correlating with PPARγ levels. ChIP assays performed in basal conditions show a ZAC enrichment in HT29 cells. In HCT116, ZAC is highly recruited at the *PPARG* promoter after epigenetic treatments correlating with *PPARG* transcription recovery *P<0.05; **P = 0.004; ***P = 0.0001. (**C**) qChIP analysis shows enrichment of MeCP2 at the *PPARG* promoter that is lost after pharmacological treatments. (**D**) A specific MeCP2-siRNA transfected into HCT116 cells determines complete silencing of its own gene and PPARγ re-expression, as assessed by Western blot, relatively to controls *P = 0.01. (**E**) qChIP analysis shows that trimethylated H3K27 is enriched in HCT116 as compared to HT29 cells. After AZA/TSA addition, H3K27 is unchanged in HT29 and reduced in HCT116 cells *P<0.05. (**F**) A specific EZH2-shRNA introduced in HCT116 efficiently silences its own gene and induces PPARγ expression, as illustrated by Western-blot analysis. This coincides with reduced H3K27me3 levels analyzed by qChIP. *P<0.05. The time-points for co-treatments were 72 hs for 5 µM AZA and 24 hs for 300 nM TSA, alone or in combination; CC indicates untreated control cells. Error bars indicate the standard deviation of the mean.

### *PPARG* silencing is associated with an increased growth rate and higher invasiveness of CRC cells

PPARγ seems to play a role in cell proliferation and invasiveness [6], [24]. To investigate whether CRC cells growth and invasiveness correlate with PPARγ levels, we compared the HCT116 and HT29 proliferation index. HCT116 showed a proliferation rate two-fold higher than HT29 cells (**Figure 5** **, panel A**). We also assessed the motility and invasiveness of the two cell lines by performing the wound-healing and migration assays. Interestingly, HCT116 showed a higher motility and invasive potential than HT29 cells (**Figure 5** **, panels B and C**). To investigate whether these HCT116 growth characteristics rely on *PPARG* expression, we stably silenced *PPARG* in HT29 cells. Among the HT29 clones tested for PPARγ levels, the clone shPPARG displayed a reduction of more than 60% than cells transfected with the empty vector or with a vector carrying non-specific shRNA (**Figure 5** **, panel D**). According to our hypothesis, the shPPARG clone showed a higher cell proliferation index, lower apoptotic rate and increased invasion potential than HT29 transfected with a non-specific shRNA (**Figure 5** **, panels E and F and Figure S4**). Regarding the apoptotic rate, administration of TZD had no effect on the HT29 shPPARG clone, as compared to parental cells (**Figure S4**). Furthermore, we generated HCT116 cells stably over-expressing a transfected wild type PPARγ (**Figure 5** **, panel G**). Consistently, in the presence of TZD these clones were inhibited in their growth and displayed a higher apoptotic index than the parental cells transfected with an empty vector (**Figure 5** **, panel H and Figure S4**). These clones showed also a reduced invasiveness and increased E-cadherin expression than the parental cells (**Figure 5** **, panels G–I**). Collectively these results suggest that *PPARG* differential expression and a TZD-dependent activity accounts for the different growth and motility properties of the CRC cell lines analyzed.

**Figure 5:** *PPARG* silencing increases proliferation and migration/invasiveness of CRC cells. (**A**) MTT assays on HCT116 and HT29 cells were carried out at different time-points *P = 0.004; **P = 0.001. (**B**) A wound-healing migration assay was carried out comparing and measuring the “wound area” at 24 and 48 hs *P = 0.045; **P = 0.0051; ***P = 0.0001. (**C**) Transwell migration assay was performed counting the run-through cells in 10 microscopic fields *P = 0.024; **P<0.01. The symbols represent the mean values of three independent experiments (mean ± SD). (**D**) Specific *PPARG*- or scrambled-shRNAs were stably transfected into HT29 cells to generate the shPPARG or control clones, respectively; the extent of PPARγ knock-down was documented by Western blot and referred to β-actin. (**E**) shPPARG cells showed higher proliferation than control clones and parental cells *P = 0.022; **P = 0.012. (**F**) The wound-healing migration and transwell migration assays were performed on the HT29 parental, the shPPARG and the control clone, respectively. The measurements were done as above. In both cases, cells were fixed after 48 hs and stained with hematoxylin & eosin or crystal violet, respectively. Magnification: 100×. Quantification of the wound-area after 24 and 48 hs is reported in the histogram where the control was set at 100%, *P = 0.016, **P = 0.001. Bars represent mean values ± SD of three independent experiments. (**G**) HCT116 cells were stably transfected with an empty expression vector or a vector carrying the PPARγ cDNA to generate control or the HCT116-PPARγ clones, respectively. Western blot analysis of the transfected PPARγ and activated target E-cadherin referred to β-actin. (**H**) The HCT116-PPARγ cells showed lower proliferation than control clones and parental cells in the presence of TZD *P = 0.012. (**I**) The wound-healing migration assay in HCT116 parental, the HCT116-PPARγ and the control clone. Cells were fixed after 48 hs and stained with hematoxylin & eosin. Magnification: 100×. The histogram shows quantification of the wound-area, measured as above, with the control set at 100%. Bars represent mean values ± SD of three independent experiments *P<0.05; **P<0.01.

## Discussion

Colorectal cancer is one of the most frequent malignancies in western countries and the third most common cause of cancer-related death worldwide [10], [13]. Among genetic alterations, chromosomal and microsatellite instability (CIN and MSI) have been invoked in CRC tumorigenesis. Several lines of evidence suggest that also epigenetic modifications contribute to the establishment and/or to the progression of a tumour [12], [13]. DNA hypermethylation is the most common epigenetic change observed in human cancers, particularly in CRC, where it is associated with TSGs silencing [12], [13]. In colorectal tumorigenesis, the precise role played by *PPARG* has been questioned because of the conflicting results reported [4]–[10]. *PPARG* mutations alone do not fully explain the frequent variations in expression detected in tumours [9], [10], [25]. Here, we provide evidence that epigenetic alterations at the *PPARG* promoter are related with gene repression that occurs in 30% of CRCs. Dissecting the *PPARG* proximal promoter, we demonstrate that a specific DNA segment (M3) is differentially methylated and *PPARG* expression is directly correlated with its methylation status (**Figs. 1** **and** **2**). Consistent with this observation, only 8% of the paired normal mucosa is methylated in the same region, probably due to the so-called “field defect” [13]. An association with patients' age at diagnosis was observed also in our CRC samples.

We also demonstrate that a reduced *PPARG* expression due to specific promoter methylation is associated with advanced tumour stages (Duke's stages C–D), deep invasion, and, ultimately, shorter survival. Other molecular alterations such as *KRAS* and *BRAF* mutations do not seem to be associated with *PPARG* methylation, while a correlation with the microsatellite instability status was found (**Figure S1**) [10]. These data imply that *PPARG* promoter methylation could be associated with CRC progression, providing a molecular basis to our previous data and to a recent proposal of *PPARG* as a favourable prognostic marker for CRC survival [9], [10]. It is poorly understood whether other genetic and epigenetic events contribute not only to *PPARG* silencing but also to overexpression detected in about 60% of CRCs. Likewise it is not clear whether this epigenetic change is a cause or a consequence of tumor progression. A subset of CRCs characterized by wide-spread methylation at CpG islands in the promoter regions of several genes is recognized as CIMP. This group appears not to be directly correlated with *PPARG* hypermethylation (our unpublished data), suggesting that methylation at this specifc gene promoter is not caused by an aberrant spread of methylation over extended genomic regions. Consistently, LINE methylation levels, a surrogate marker of global DNA methylation, does not correlate with *PPARG* expression in CRC [10]. It is worth of note that methylation at the M3 segment of the *PPARG* promoter occurs not only in tumours *in vivo* but also in CRC derived cell lines. This is the first report that shows promoter methylation to play a role in *PPARG* repression in tumorigenesis. The only analysis reported so far, refers to the *Pparg*2 promoter in a mouse model of diabetes related to the adult metabolic syndrome [26]. The results obtained in 3T3-L1 preadipocytes and extended to the human gene, for structure and sequence similarities, suggest that also *PPARG*2 is regulated by DNA methylation [26]. More recently, epigenetic regulation of *Pparg* has been invoked as an important step in mouse myofibroblast transdifferentiation of hepatic stellate cells that promotes liver fibrogenesis [22].

The link between DNA methylation and histone modifications is mediated by a group of proteins with methyl-CpG-binding activity. MeCP2 recruits co-repressor complexes including HDACs and HMTs [27]. Its role in tumorigenesis is, however, still debated [22], [27], [28]. EZH2 is also recruited and appears to be involved in the maintenance of the repressed status [21]. Both MeCP2 and EZH2 have recently been shown to be key regulators of *Pparg* repression [22]. Consistently, MeCP2 and EZH2 levels inversely correlate with *PPARG* expression in the CRC cells investigated. In the silenced state, as in *PPARG-*negative HCT116 cells, the promoter is significantly enriched in HDAC1, MeCP2 and chromatin repressive marks such as H3K9me3 and H3K27me3. This latter suggests the presence of EZH2-containing repressive complexes. Differently, exposure to AZA and TSA causes replacement with active chromatin marks such as H3K9Ac and H3K4me3, accompanied by a complete loss of HDAC1 and MeCP2. Recruitment of RNAPol-II and P-RNAPol-II under these conditions fully correlates with the ability of the newly synthesized receptor to transactivate a reporter gene. MeCP2 and EZH2 silencing re-activate PPARγ, confirming their crucial role in *PPARG* epigenetic repression. These conclusions are supported by the enhanced growth properties of HT29 cells carrying a silenced *PPARG* and by the reduced growth rate and migration properties of HCT116 over-expressing a transfected wild type PPARγ. Collectively these functional analyses suggest that *PPARG* silencing may actively contribute to colon tumor progression. Thus, we propose a novel regulatory model in which an unmethylated (or partially methylated) *PPARG* core promoter region is normally recognized by unknown transcriptional activators, among which only the zinc-finger protein ZAC has been identified so far in CRC cells [23]. Upon promoter methylation, HDAC1 and MeCP2 repressive complexes are recruited to form a condensed chromatin structure that suppresses transcription initiation. In this context, EZH2-containing repressive complexes are further recruited, fully “marking” the histones via H3K27 methylation to establish a stable *PPARG* silencing by blocking transcription elongation (**Figure 6**). *PPARG* has been shown to potentiate the effects of a variety of chemotherapeutic regimens on the assumption that the addition of a specific ligand would render the receptor more efficient in transactivating target genes [29]. Only few evidences in the literature support the notion of adding a specific PPARγ agonist to well-established chemotherapeutic regimens for the treatment of *PPARG*-positive CRCs [30]. On the basis of our data, it is tempting to speculate a possible intervention for the treatment of *PPARG*-negative CRCs, based on the combination of a conventional chemotherapy with epigenetic drugs and a specific PPARγ agonist [31]. This regimen would re-establish PPARγ expression and activity, sensitize the tumour to the therapy, overcome possible resistance to the agonist and result in a better outcome with possibly longer survival.

**Figure 6:** Schematic drawing of the proposed molecular mechanism(s) of *PPARG* silencing. (**I**) The unmethylated or partially methylated *PPARG* core promoter is activated by unknown transcriptional factors, among which only the zinc-finger protein ZAC that induces apoptosis and cell-cycle arrest has been identified. (**II**) Upon extensive promoter DNA methylation, MeCP2, HDAC1 and EZH2 containing repressive complexes are recruited to form a condensed chromatin structure, inhibiting RNA polymerase II and impairing gene transcription.

In conclusion, we demonstrate that epigenetic events play a role in *PPARG* expression. DNA methylation and the associated chromatin repressive marks are responsible for *PPARG* silencing in a proportion of sporadic CRCs and derived cell lines. Larger epidemiological studies are required to support this hypothesis and to translate these results into clinical practice.

## Supporting Information

Figure S1 Correlation between K-RAS and B-RAF mutations, microsatellite instability and PPARG methylation in CRCs. A subset of our colorectal cancer series was analyzed for K-RAS mutations at codons 12, 13 and B-RAF mutation at codon 600. CRCs were stratified based on Microsatellite stability (MSS) or instability (MSI) and related to PPARG methylation status (in grey).
(2.85 MB TIF)

Figure S2 Loss of PPARG expression in CRC cell lines is due to DNA promoter methylation. (A) PPARG Loss Of Heterozigosity (LOH) was tested in HCT116 and HT29 cells using two DNA markers flanking the PPARG locus at the 5′ and 3′ end, respectively. No differences were appreciated, indicating that the locus had not been rearranged. Size marker = SM. (B) Activation of the MAPK/ERK signalling pathway did not correlate with the loss of PPARG expression. Basal and phosphorylated ERK levels were lower in PPARG-negative HCT116 than in PPARG-positive HT29 cells. (C) Quantitative ChIP analysis demonstrated enrichment of 5-methyl-cytosine (5-MeC) at the PPARG promoter in HCT116 with respect to HT29 cells. Epigenetic treatment significantly reduced 5-methyl-cytosine only in HCT116 cells *P<0.01. Error bars indicate the standard deviation of the mean.
(1.90 MB TIF)

Figure S3 Synergistic effect of AZA and Trichostatin A (TSA) on PPARG re-activation. (A) HCT116 were treated with 1- 5 μM AZA for 72 hs, with 300 nM TSA for 24 hs alone or in combination with 1 or 5 μM AZA. HT29 cells served as control. PPARγ levels were analyzed by western-blot and quantified referring to β-actin. The histograms show that AZA/TSA in combination induce a synergistic PPARG re-activation only in HCT116 cells *P<0.05, **P<0.01, ***P = 0.0001, whereas no significant differences were observed in treated HT29 as compared to untreated control cells. (B) To confirm the synergistic effect on PPARγ activity, HCT116 were treated with AZA and TSA alone or in combination and transiently transfected with the PPRE-TK-luciferase reporter gene. After twelve hours the cells were treated with 1μM TZD or GW9662, a selective antagonist, or the vehicle alone (V). TZD administration increased the luciferase reporter gene activity, while exposure to GW9662 drastically reduced it even if compared with the vehicle alone. Luciferase activity was determined and normalized to β-galactosidase for transfection efficiency. Results are the mean values ± SD of three independent experiments, each performed in duplicate and compared with the corresponding controls; CC indicates untreated control cells *P<0.01; **P = 0.002.
(2.61 MB TIF)

Figure S4 HDAC1, MeCP2 and EZH2 expression levels in CRCs samples and cell lines. (A) Western blot analysis for HDAC1 was carried out in HCT116 and in the indicated CRC cell lines. (B) Protein extracts from representative tumour tissues (T) and matched adjacent normal mucosa (N) were analyzed for HDAC1, EZH2 and MeCP2. β-actin was used as internal control in both cases. (C) Immunohistochemical analysis of some representative tumour samples expressing high and low HDAC1 and PPARγ levels, respectively. (D) HDAC1, EZH2 and MeCP2 expression levels in a subset of CRCs (N = 20) and paired normal mucosa are represented by box-plot. The edges of the boxes are the interquartile range box, lines in the boxes represent the median value; the P value in each graph was obtained by the Mann-Whitney test (E). In some representative tumour samples (n = 52), HDAC1 and EZH2 high expression was directly related with C-D Duke's tumour stages. The same relationship was not found for MeCP2. P value was calculated by the Spearman correlation. (F) To assess the apoptotic rate induced by the PPARγ ligand troglitazone (TZD), flow cytometrical analysis (FCA) was carried out in HT29 parental cells transfected with a control plasmid (CC) or with an shPPARG. Alternatively, FCA was performed in HCT116 transfected with an empty vector (EV) or with an expression vector for PPARγ HCT116+PPARGγ.
(1.24 MB PDF)

Table S1 (0.05 MB DOC)

Table S2 (0.04 MB DOC)
